The article "Identification and Classification of Enhancers Using Dimension Reduction Technique and Recurrent Neural Network" was published in 2020. Journal: Comput Math Methods Med.

# Identification and Classification of Enhancers Using Dimension Reduction Technique and Recurrent Neural Network

**DOI:** 10.1155/2020/8852258

**Published:** 2020-10-18

**Authors:** Qingwen Li, Lei Xu, Qingyuan Li, Lichao Zhang

**Affiliations:** ^1^College of Animal Science and Technology, Northeast Agricultural University, Harbin, China; ^2^Institute of Fundamental and Frontier Sciences, University of Electronic Science and Technology of China, Chengdu, China; ^3^School of Electronic and Communication Engineering, Shenzhen Polytechnic, Shenzhen, China; ^4^Forestry and Fruit Tree Research Institute, Wuhan Academy of Agricultural Sciences, Wuhan, China; ^5^School of Intelligent Manufacturing and Equipment, Shenzhen Institute of Information Technology, Shenzhen, China

## Abstract

Enhancers are noncoding fragments in DNA sequences, which play an important role in gene transcription and translation. However, due to their high free scattering and positional variability, the identification and classification of enhancers have a higher level of complexity than those of coding genes. In order to solve this problem, many computer studies have been carried out in this field, but there are still some deficiencies in these prediction models. In this paper, we use various feature extraction strategies, dimension reduction technology, and a comprehensive application of machine model and recurrent neural network model to achieve an accurate prediction of enhancer identification and classification with the accuracy of was 76.7% and 84.9%, respectively. The model proposed in this paper is superior to the previous methods in performance index or feature dimension, which provides inspiration for the prediction of enhancers by computer technology in the future.

## 1. Introduction

Enhancers are a small area of DNA that can link with protein, located upstream or downstream of the gene, and gene transcription will be enhanced after they bind with protein [1]. Because of the winding structure of chromatin, enhancers being far apart in the sequence still have the opportunity to contact each other. Therefore, they are not necessarily close to the gene to be affected, or even located on the same chromosome as the gene. Studies have shown that enhancer mutations may lead to a variety of diseases.

Owing to the significance of enhancers, the identification and classification of enhancers have always been the focus of computational biologists and experimental biologists [2, 3]. The fact is that to identify enhancers by biochemical experiments is expensive and time-consuming.

In the past few years, some bioinformatics methods have been developed to predict enhancers [4]. Liu et al. [5] proposed iEnhancer-2L, which extracts features by pseudo *k*-tuple nucleotide composition and achieves the enhancer identification and classification with the accuracy of 73% and 60.5%, respectively. Jia and He [6] suggested EnhancerPred, which extracts features by biprofile Bayes and pseudo *k*-tuple nucleotide composition to support the vector machine and achieves the accuracy of 75% and 55% for the prediction of enhancer identification and classification, respectively, Liu et al. [7] proposed iEnhancer-EL, which applies K-mer, pseudo *k*-tuple nucleotide composition and subsequence profile feature extraction methods and uses the ensemble classifier based on support vector machine to achieve the accuracy of 74.8% for enhancer identification and 61% for enhancer classification [8]. Nguyen et al. [9] proposed iEnhancer-ECNN, which uses a convolutional neural network to achieve the accuracy of 76.9% for enhancer identification and 67.8% for enhancer classification prediction [10]. All of the above methods emphasize the better prediction results but fail to mention the dimensional advantages of the model [11, 12]. Due to the fact that high-dimensional features may lead to an over-fitting and high-dimension disaster or an increase of redundant information, the machine learning model trained by this initial high-dimension feature is often found to be underperforming in practice [13–17].

The article "Identification and Classification of Enhancers Using Dimension Reduction Technique and Recurrent Neural Network" was published in 2020. Journal: Comput Math Methods Med.

In this paper, a low dimensional feature model is obtained by using a variety of feature extraction strategies and dimension reduction technology [18–23]. The identification and classification of enhancers have been achieved via the combination of machine learning models and artificial neural network with the accuracy rate of 76.7% and 84.9%, respectively. It also should be noted that the dimension of the feature model used to identify enhancers is only 37, which is much lower than the past methods. And this paper also got an 18-dimension feature model for enhancer identification, and its accuracy reached 76.5% after testing.

## 2. Materials and Methods

In this paper, the identification and classification of enhancers are described by Figures 1 and 2, respectively.

### 2.1. Benchmark Dataset

This paper used a dataset proposed by Liu et al., which was also used in the development of iEnhizer-2L, EnhancerPred, iEnhancer-EL, and iEnhancer-ECNN. In this dataset, enhancer information was collected from 9 different cell lines, and DNA sequences of 200 bp in length were extracted. In order to avoid the deviation of the classifier, enhancers with the similarity of over 90% were deleted from the dataset through CD-HIT [24, 25]. The dataset contains 1484 enhancers and 1484 nonenhancers. Among them, 1484 enhancers include 742 strong enhancers and 742 weak enhancers.

The article "Identification and Classification of Enhancers Using Dimension Reduction Technique and Recurrent Neural Network" was published in 2020. Journal: Comput Math Methods Med.

### 2.2. Feature Extraction

Machine learning algorithms cannot directly perform annotations on continuous nucleotide sequences, so it is necessary to convert nucleotide sequences represented by strings into feature vectors represented by numbers [26–28]. This paper implemented feature extraction through iLearn [29].

#### 2.2.1. K-mer

The K-mer feature extraction strategy refers to calculating the frequency of the unit in the entire sequence with k adjacent nucleotides as a unit [30, 31]. This paper uses 1-mer, 2-mer, 3-mer, and 4-mer feature extraction methods, which are stated by the following formulas:

(1) $$\begin{array}{c} 1-\text{mer}:f\left(a\right)=\frac{N_{a}}{N_{t}},a\in \left(\text{A},\text{T},\text{C},\text{G}\right),\\ 2-\text{mer}:f\left(a,b\right)=\frac{N_{a}}{\left(N_{t}-1\right)},a,b\in \left(\text{A},\text{T},\text{C},\text{G}\right),\\ 3-\text{mer}:f\left(a,b,c\right)=\frac{N_{abc}}{\left(N_{t}-2\right)},a,b,c\in \left(\text{A},\text{T},\text{C},\text{G}\right),\\ 4-\text{mer}:f\left(a,b,c,d\right)=\frac{N_{abcd}}{\left(N_{t}-3\right)},a,b,c,d\in \left(\text{A},\text{T},\text{C},\text{G}\right). \end{array}$$

*N*_*t*_ is the length of a DNA sequence and *N*_*a*_, *N*_*ab*_, *N*_*abc*_, *N*_*abcd*_ are the units composed of adjacent K nucleotides.

#### 2.2.2. Reverse Compliment K-mer (RCK-mer)

Reverse Compliment K-mer is a variant of K-mer, which ignores the complementary sequences of adjacent nucleotide sequences. For example, there are 16 types of 2-mer: “AA,” “AC,” “AG,” “AT,” “CA,” “CC,” “CG,” “CT,” “GA,” “GC,” “GG,” “GT,” “TA,” “TC,” “TG,” and “TT.” Because ‘TT' is the reverse completion K-mer of “AA,” it can be left out. Therefore, there are only 10 kinds of 2-mer in this method: “AA,” “AC,” “AG,” “AT,” “CA,” “CC,” “CG,” “GA,” “GC,” and “TA.” The frequency of each K-mer was calculated in turn.

#### 2.2.3. Enhanced Nucleic Acid Composition (ENAC)

Enhanced nucleic acid composition is the frequency of each nucleotide occurring within a fixed sequence window length, which slides continuously from the 5′ end to the 3′ end of each nucleotide sequence and usually used to encode nucleotide sequences of the same length.

#### 2.2.4. Composition of K-Spaced Nucleic Acid Pairs (CKSNAP)

This method calculated the frequency of pairs of nucleotides separated by K nucleotides in the whole sequence. When *k* = 0, it is consistent with the features represented by 2-mer. It should be noted that the frequency of nucleotide pairs is calculated though, when *k* = 0, 1, 2, 3, 4, and 5, the length of sequences should be L-1, L-2, L-3, L-4, L-5, and L-6.

The article "Identification and Classification of Enhancers Using Dimension Reduction Technique and Recurrent Neural Network" was published in 2020. Journal: Comput Math Methods Med.

#### 2.2.5. Nucleotide Chemical Property (NCP)

The method took into account different chemical structures and chemical properties of four nucleotides [32, 33]. “A” is presented as (1, 1, 1), “C” as (0, 1, 0), “G” as (1, 0, 0), and “T” as (0, 0, 1).

#### 2.2.6. Accumulated Nucleotide Frequency (ANF)

This method combined the approach of nucleotide chemical properties and considers the chemical properties, the location, and the frequency of each nucleotide. For example, for a sequence “TCGTTCATGG,” “T” appears in bits 1, 4, 5, and 8, with frequencies corresponding to 1 (1/1), 0.5 (2/4), 0.6 (3/5), and 0.5 (4/8), respectively; “C” appears in bits 2 and 6, with frequencies corresponding to 0.5 (1/2) and 0.33 (2/6), respectively; “G” appears in bits 3, 9, and 10, with frequencies corresponding to 0.33 (1/3), 0.22 (2/9), and 0.3 (3/10), respectively; “A” appears in the 7th position, so its frequency was 0.14 (1/7). Therefore, the sequence can be expressed as {(0, 0, 1, 1), (0, 1, 0, 0.5), (1, 0, 0, 0.33), (0, 0, 1, 0.5), (0, 0, 1, 0.6), (0, 1, 0, 0.33), (1, 1, 1, 0.14), (0, 0, 1, 0.5), (1, 0, 0, 0.22), (1, 0, 0, 0.3)} [34, 35].

#### 2.2.7. Electron-Ion Interaction Pseudopotentials of Trinucleotide (EIIP)

Nair and Pillai [36] proposed the Electron-Ion Interaction Pseudopotentials of Trinucleotide (EIIP) of nucleotides A, G, C, and T. The EIIP of the four nucleotides is A: 0.1260, C: 0.1340, G: 0.0806, and T: 0.1335. This method directly used the EIIP to represent the nucleotides in the DNA sequence. Therefore, the dimension of EIIP is the length of the DNA sequence.

#### 2.2.8. Electron-Ion Interaction Pseudopotentials of Trinucleotide (PseEIIP)

In these codes, EIIPA, EIIPT, EIIPG, and EIIPC were used to represent the EIIP of nucleotides A, T, G, and C, respectively. Then, the average value of EIIP of the three nucleotides in each sample was used to construct the feature vector, which can be expressed as follows:

(2) $$\begin{array}{c} V={\left[{\text{EIIP}}_{\text{AAA}}\times f_{\text{AAA}},{\text{EIIP}}_{\text{AAC}}\times f_{\text{AAC}},{\text{EIIP}}_{\text{AAG}}\times f_{\text{AAG}},\cdots ,{\text{EIIP}}_{\text{TTG}}\times f_{\text{TTG}},{\text{EIIP}}_{\text{TTT}}\times f_{\text{TTT}}\right]}_{64}. \end{array}$$

*f*_*abc*_, *a*, *b*, *c* ∈ (A, T, C, G) is the normalized frequency of a trinucleotide, and EIIP_*abc*_, *a*, *b*, *c* ∈ (A, T, C, G) is the sum of EIIP values of three nucleotides.

#### 2.2.9. One-Hot

Each enhancer in the dataset is a 200 bp nucleotide sequence, which consists of four nucleotides, namely, adenine (A), guanine (G), cytosine (C) and thymine (T). Each nucleotide is represented by a set of vectors (Table 1) [37, 38].

The article "Identification and Classification of Enhancers Using Dimension Reduction Technique and Recurrent Neural Network" was published in 2020. Journal: Comput Math Methods Med.

### 2.3. Feature Selection

Feature selection is the method of selecting a subset of related features used in model construction [39, 40]. Because the dimension of features will be reduced after selection, this process is called dimension reduction.

#### 2.3.1. MRMD2.0

This paper used MRMD2.0 [41] to achieve dimension reduction. Firstly, MRMD2.0 uses seven main feature ranking methods (ANOVA, MRMD, MIC, Lasso, mRMR, chi-square test, and RFE) to calculate the feature sets, respectively, and then uses the idea of the PageRank algorithm to comprehensively process the results of the seven feature ranking algorithms and get the final feature ranking, Then, using the positive addition strategy, the features arranged in descending order are added to the feature subset for verification, and the best feature subset is finally obtained.

#### 2.3.2. Evolutionary Search

Evolutionary Search uses evolutionary algorithms for feature selection. An evolutionary algorithm is not a specific algorithm; it includes a variety of algorithms (genetic algorithm, memetic algorithm, and multiobjective evolutionary algorithm). The inspiration of the evolutionary algorithm draws on the evolutionary operations of living things in nature. Compared with traditional optimization algorithms such as calculus-based methods and exhaustive methods, it is a mature global with high robustness and wide applicability. The optimization method has the characteristics of self-organization, self-adaptation, and self-learning. It is not limited by the nature of the problem and can effectively handle complex problems that are difficult to solve by traditional optimization algorithms.

### 2.4. Classifier

#### 2.4.1. Recurrent Neural Network

This paper also used recurrent neural networks to make predictions on the basis of the memory model. It is expected that the network can remember the previous features and infer the subsequent results according to the features; hence, the overall network structure continues in the cycle. The biggest problem with memory is that it has forgetfulness. We can always remember the recent events more clearly and forget the events that happened long ago. Recurrent neural networks also have this problem. In order to solve this problem, two variants of the network structure have emerged: one is called LSTM, and the other is called GRU. Both of these variants can well solve the problem of long-term dependence.

#### 2.4.2. Random Forest

In this study, a random forest was applied to play a role as a classifier for prediction. Random forest is widely employed in the bioinformatics research [42–52]. This classifier concludes multiple decision trees while the output category is arranged by the mode of the category output by trees individually. This paper implemented a random forest classifier through the weka platform.

The article "Identification and Classification of Enhancers Using Dimension Reduction Technique and Recurrent Neural Network" was published in 2020. Journal: Comput Math Methods Med.

#### 2.4.3. Support Vector Machine

As a very powerful machine learning method widely used in biological sequence prediction [53–71], the support vector machine was used for prediction in this research. It is a class of generalized linear classifiers that classify data binary in a supervised learning method, and its decision boundary is the maximum margin hyperplane that is solved for the learning sample. This paper used libSVM to implement support vector machine and adjust parameters *c* and *g* using grid to optimize the prediction results.

#### 2.4.4. libD3C

This paper also applied the libD3C classifier [72] to test the performance of models. The classifier adopts a selective ensemble strategy, based on the hybrid ensemble pruning model combining *k*-means clustering and function selection cycle framework and sequential search, by training multiple candidate classifiers and then selecting a set of accurate and different classifiers to settle the problem.

### 2.5. Evaluation of Prediction

This paper used sensitivity (Sn), specificity (Sp), total accuracy (Acc), and Mathew (Mcc) correlation coefficients to evaluate the performance of the model [73–83].

(3) $$\begin{array}{c} \text{Sn}=\frac{\text{TP}}{\left(\text{TP}+\text{FN}\right)},\\ \text{Sp}=\frac{\text{TN}}{\left(\text{TN}+\text{FP}\right)},\\ \text{Acc}=\frac{\left(\text{TP}+\text{TN}\right)}{\left(\text{TP}+\text{TN}+\text{FP}+\text{FN}\right)},\\ \text{Mcc}=\frac{\left(\text{TP}\times \text{TN}-\text{FP}\times \text{FN}\right)}{\sqrt{\left(\text{TP}+\text{FP}\right)\times \left(\text{TP}+\text{FN}\right)\times \left(\text{TN}+\text{FP}\right)\times \left(\text{TN}+\text{FN}\right)}}. \end{array}$$

TP is true positive; FN is false negative; FP is false positive; TN is true negative.

## 3. Results and Discussion

### 3.1. Identification of Enhancers

Feature vectors of enhancers and nonenhancers were obtained by K-mer, RCK-mer, ENAC, CKSNAP, NCP, ANF, EIIP, PseEIIP, and One-Hot feature extraction methods. In order to determine which feature extraction methods were suitable for the identification of enhancers, the random forest was adopted through ten-fold cross-validation for each method. After testing (Figure 3), this paper believed that 2-mer, 3-mer, 4-mer, CKSNAP, ENAC, PseEIIP, and RCK-mer, the seven feature extraction methods, were more effective. Since the dimension of the feature model obtained through the seven extraction methods was rather high, which could cause the classifier overfitting the training set and lead to a less effective performance in practical applications. This paper expected to get a low-dimension and excellent performance feature model; hence, the seven feature models were merged after individual dimension reduction through MRMD2.0; then, we found that the dimension was 1049, which was still relatively high. Therefore, the merged model went through 5 consecutive dimension reductions by MRMD2.0, and a 37-dimension feature model was achieved eventually. At this time, the dimension can no longer be reduced further (Figure 4). Using the random forest classifier, the 37-dimension feature model was tested through ten-fold cross-validation (Table 2), and the accuracy reached 76.7%; the running time of the method is 2.14 seconds.

The article "Identification and Classification of Enhancers Using Dimension Reduction Technique and Recurrent Neural Network" was published in 2020. Journal: Comput Math Methods Med.

At the same time, this paper used Evolutionary Search to reduce the dimension of the merged 1049-dimensional model to compare the differences between different dimension reduction tools. After 8-dimension reductions, an 18-dimension model was obtained in this paper, and the accuracy rate reached 76.5% after 10-fold cross-validation. Although this feature model is inferior to the model obtained by MRMD2.0 in performance, it has obvious advantages in dimension. The 18-dimensional feature model may imply that it is an important marker for distinguishing enhancers. These 18-dimension features come from 4-mer, 2-mer, CKSNAP, RCK-mer, and PseEIIP, respectively, indicating that specific dinucleotides, trinucleotides, and their electronic-ion interactions play an important role in enhancer sequences. By using two tools, we can find that Evolutionary Search has an advantage in dimension after dimension reduction, and MRMD2.0 has more advantages in terms of performance parameters after dimension reduction.

In order to further determine the stability of the feature model, this paper used support vector machine and libD3C to test the 37-dimension model at the same time (Table 2). Through the support vector machine combined with the grid search method (c 8192.0, g 0.001953125), the accuracy reached 76.5%. Using the libD3C classifier, the accuracy reached 75.5%. The prediction accuracy of the three classifiers for the feature model all exceeded 75%, indicating a very stable feature model. Meanwhile, in addition to the excellent performance of the feature model examined in this paper, it also has a very low dimension compared with a previous work (Table 2), which can effectively avoid dimensional disasters.

### 3.2. Classification of Enhancers

For the feature extraction of strong enhancers and weak enhancers, the same methods as enhancer identification were adopted, and then, the random forest was used through ten-fold cross-validation to examine the performance. After testing, this paper believed that also 2-mer, 3-mer, 4-mer, CKSNAP, ENAC, PseEIIP, and RCK-mer, the seven feature extraction methods, perform slightly better than other methods, but were not satisfactory. Therefore, this paper attempted to improve accuracy through dimension reduction techniques. After reducing the dimensions of the seven feature models that performed slightly better, they were merged to continue the dimension reduction. After four dimension reductions, an 82-dimension feature model was obtained. At this time, it was impossible to continue the further dimension reduction. The 82-dimension model was cross-validated with a random forest classifier, and the accuracy of 62.3% was still not ideal.

The article "Identification and Classification of Enhancers Using Dimension Reduction Technique and Recurrent Neural Network" was published in 2020. Journal: Comput Math Methods Med.

Next, this paper used the voting mechanism to output the prediction results of the 82 feature model of the three classifiers libSVM, random forest, and libD3C and retained the prediction results with the highest confidence based on the given confidence of each classifier result. After statistics, the final accuracy was 63.1%, the result was still not ideal.

As the recurrent neural network has contributed a lot in the fields of sequence problems and natural language processing with a limited capacity of memory, the variant of recurrent neural network—Long Short-Term Memory—was applied in this research to predict biological sequences. This paper used the 3-mer method to segment the sequence and then trained the word embedding through word to vector. Next, this study used the LSTM model based on the attention mechanism to predict the word segmentation file. When the model was a two-layer neuron, hidden_dim was 100, the learning rate was 0.005, and the adam optimizer was used; the accuracy of ten-fold cross-validation reached 84.9%. After comparison (Table 3), this paper has achieved ideal results in the classification of enhancers.

## 4. Conclusions

In this paper, a 37-dimension feature model for identifying enhancers was obtained through multiple dimension reductions. After testing, the performance of the model was sound and stable. At the same time, this paper has achieved ideal results in the classification of enhancers through 3-mer methods, word to vector techniques, and RNN models. It is expected that the method proposed in this paper can provide a certain reference for the future research on enhancers in the academic world.

## Figures and Tables

**Figure 1:** Research process of enhancer identification.

**Figure 2:** Research process of enhancer classification.

**Figure 3:** (a) The accuracy of different feature extraction methods after verification. Through analysis, this article believed that the method represented by dark blue had higher accuracy, while the method represented by purple had lower accuracy. (b) Changes in accuracy of different extraction methods before and after dimensionality reduction. Through analysis, this paper believed that accuracy has improved after dimensionality reduction.

The article "Identification and Classification of Enhancers Using Dimension Reduction Technique and Recurrent Neural Network" was published in 2020. Journal: Comput Math Methods Med.

**Figure 4:** The relationship between accuracy change and dimension change. According to trends, this paper believed that dimension and accuracy are negatively correlated. Using MRMD2.0, when the dimension was 37, the accuracy reached 76.68%, and the dimension reduction continued; the accuracy cannot be improved.

**Table 1:** One-Hot encoding.

Nucleotides	Code
A	[1,0,0,0]
T	[0,0,0,1]
C	[0,1,0,0]
G	[0,0,1,0]

**Table 2:** The comparison between this paper and the previous work on enhancer identification.

	Acc	AUC	SN	SP	MCC	Dimension
iEnhancer-2L	0.730	0.806	0.710	0.750	0.460	
EnhancerPred	0.740	0.801	0.735	0.745	0.480	
iEnhancer-EL	0.748	0.817	0.710	0.785	0.496	
iEnhancer-ECNN	0.769	0.832	0.785	0.752	0.537	2400
Our method	0.767	0.837	0.733	0.801	0.535	37

**Table 3:** The comparison between this paper and the previous work on enhancer classification.

	Acc	SN	SP	MCC
iEnhancer-2L	0.605	0.470	0.740	0.218
EnhancerPred	0.550	0.45	0.65	0.102
iEnhancer-EL	0.61	0.540	0.68	0.222
iEnhancer-ECNN	0.678	0.791	0.564	0.368
Our method	0.849	0.858	0.84	0.699

## Data Availability

The raw data supporting the conclusions of this article will be made available by the authors, without undue reservation.
